# Cementless Hydroxyapatite Coated Hip Prostheses

**DOI:** 10.1155/2015/386461

**Published:** 2015-02-23

**Authors:** Antonio Herrera, Jesús Mateo, Jorge Gil-Albarova, Antonio Lobo-Escolar, Elena Ibarz, Sergio Gabarre, Yolanda Más, Luis Gracia

**Affiliations:** ^1^Department of Surgery, Medicine School, University of Zaragoza, Domingo Miral s/n, 50009 Zaragoza, Spain; ^2^Aragón Health Sciences Institute, Avenida San Juan Bosco 13, 50009 Zaragoza, Spain; ^3^Department of Orthopaedic Surgery and Traumatology, Miguel Servet University Hospital, Avenida Isabel la Católica 3, 50009 Zaragoza, Spain; ^4^Department of Orthopaedic and Trauma Surgery, San Jorge Hospital, Avenida Martínez de Velasco 36, 22004 Huesca, Spain; ^5^Department of Mechanical Engineering, Engineering and Architecture School, University of Zaragoza, María de Luna 3, 50018 Zaragoza, Spain

## Abstract

More than twenty years ago, hydroxyapatite (HA), calcium phosphate ceramics, was introduced as a coating for cementless hip prostheses. The choice of this ceramic is due to its composition being similar to organic apatite bone crystals. This ceramic is biocompatible, bioactive, and osteoconductive. These qualities facilitate the primary stability and osseointegration of implants. Our surgical experience includes the implantation of more than 4,000 cementless hydroxyapatite coated hip prostheses since 1990. The models implanted are coated with HA in the acetabulum and in the metaphyseal area of the stem. The results corresponding to survival and stability of implants were very satisfactory in the long-term. From our experience, HA-coated hip implants are a reliable alternative which can achieve long term survival, provided that certain requirements are met: good design selection, sound choice of bearing surfaces based on patient life expectancy, meticulous surgical technique, and indications based on adequate bone quality.

## 1. Introduction

Since Charnley's first design of low friction arthroplasty which emerged in the 1960s [1] a number of improvements have gradually arisen, affecting design, materials, primary and secondary implant fixation systems, and biomechanical and biological adaptations which occur in the bone after joint replacement. The main objective in all instances has been to improve the survival of the implant in the long term [2], a goal shared by all surgeons. Implant to bone fixation was initially achieved by means of acrylic cement, which was also introduced by Charnley. Although long-term outcomes of cemented hip arthroplasty have been good and modern cementing techniques can improve implant survival even further, cemented hip implants have always been a concern in young and more active patients. Cementless hip arthroplasty emerged at the end of the 1970s, as an alternative to cemented systems. Primary fixation of cementless designs is based on a tight press-fit of the implant into the bone, and secondary or definitive fixation depends on a biological anchoring in bone, needed to ensure long-term survival of the implant [3]. In early cementless designs biological fixation was poor, and loosening was common. Primary bone-implant stability is critical because although 50 to 150 *μ*m wide micromovements still allow new bone formation [4–7], the greater the magnitude of micromovements, the lower the amount of bone formation. Thus, bone-implant anchorage could turn into a fibrous tissue which leads to loosening.

In the late 1970s, porous coatings were added to implant surfaces in order to improve osseointegration [8–12]; however, a high incidence of thigh pain, bead shedding, and loosening was found. Implant osseointegration of these designs took a long time, and surgical technique was demanding. Further research on porous coatings [13] brought improvements in manufacturing which immediately improved clinical outcomes.

The search for a type of coating capable of enhancing implant osseointegration led to growing interest in calcium phosphate ceramics, which were first used for coating dental implants and then were brought into the orthopaedics field. Hydroxyapatite (HA) was chosen from calcium phosphate ceramics for its chemical characteristics and for being a major component of bone mineral content. The Leiden Biomaterials Research Group, Gloot and Geesing [14, 15], Furlong [16], Manley [17], and Epinette [18] pioneered the orthopaedic use of HA, as an osteoconductive material which promotes osseointegration of implants improving their long-term survival. Currently, HA-coated implants have been in use for nearly 30 years with excellent results. 

*Hydroxyapatite: Structure and Properties*. Synthetic calcium phosphate ceramics have similar chemical and crystalline properties to biological apatite crystals. Among them, the HA (Ca_10_(PO_4_)_6_(OH)_2_) is the most similar to biological apatite crystals, but its atomic ratio is 1.67 times greater than that of bone or dentine, and it is the least soluble of all calcium phosphate ceramics [19]. HA is biocompatible (it does not cause toxic or inflammatory responses in vivo) [20], bioactive, and osteoconductive, but HA is not osteoinductive [19]. Its mechanical characteristics include high compressive strength (700 MPa) but low tensile (250 MPa) and fatigue strength [21]. HA is used for creating a coating on prosthetic cup or stem surfaces, which are usually made of a titanium alloy (TiAlV). HA deposition is often achieved through the plasmaspray technique, which is performed at high temperature (15000°) and under vacuum, by projecting HA particles onto the metallic material at a speed of 300 m/s. The metallic substrate has a rough surface to promote adhesion. The other manufacturing method achieves HA deposition by electrochemical means, although it appears that the plasma spray technique is associated with improved bone ongrowth [22]. Advisable HA coating thickness is 50 *μ*m because coats 15–20 *μ*m thick are quickly dissolved, and coats 100–150 *μ*m thick may suffer delamination as a result of the tensile forces produced in uploading [21], even though good results have been reported with thicker (200 microns) coatings [16]. HA coating should have pores of about 100–200 microns and an acceptable porosity index to promote osteoconductivity, although coating strength decreases with porosity [19]. Another key characteristic of HA coating is crystallinity, which is associated with increased bioactivity and bone growth and with decreased bone resorption [23].

Other important matters are the HA coating resorption after implantation, or the coating delamination process, most likely in thicker coatings (150–200 microns) and unstable implants [24].

No strong evidence can be found in literature about the HA resorption process and loss of HA coating. However, two phases in HA loss have been suggested [25]. The first one, in the immediate postoperative period, is when micromovements in the HA-bone interface lead to the formation of a fibrous membrane with high metabolic activity, containing fibroblasts and macrophages which are able to remove the HA coating. This inflammatory response, described as transient by Geesink et al. [21], along with an increased fluid content and a low pH, helps to dissolve the less crystalline HA, releasing calcium ions which may have biological activity [19]. These calcium ions can be incorporated into the remaining HA coating, increasing its crystallinity and thus reducing the subsequent coating loss, which takes years to disappear [26]. The bone around the implant is also undergoing a remodeling process, adaptive remodeling, regulated by biomechanical changes, among other factors. Osteoclastic activity linked to adaptative remodeling contributes to HA resorption [19, 26–31], which is related to the thickness of the coating layer [28]. Later the lost HA coating is replaced by new bone [26–31] leading to implant osseointegration. New bone apposition on the HA coating surface begins at third postoperative week [21, 32–34], and initially it has a lamellar structure which is gradually replaced by a Haversian structure as remodeling progresses [21].

## 2. Materials and Methods

In 1990 our department started using cementless HA-coated hip implants, in particular the ABG I prosthesis (Stryker). It consists of an anatomical HA-coated stem with press-fit metaphyseal fixation and an HA-coated hemispherical cup. The ABG I implant is made of a titanium alloy (Ti6Al4V) with Young's modulus of 110 GPa (Figure 1(a)). The HA coating, applied through a plasma spraying process, was 50 *μ*m thick and of about 80% crystallinity after the manufacturing process. Until September 1999, this design was implanted in 1637 patients (bilateral in 277 of them), with a total of 1914 hip arthroplasties. The bearing surfaces were conventional polyethylene with metal or zirconia heads in all cases. In 1999, the ABG I system was replaced by a new design, the ABG II model (Figure 1(b)). The new cup has only five holes through which spikes or screws can be inserted for proper primary fixation, and hole plugs are supplied for sealing unused holes. The “shoulder” of the stem is higher and its metaphyseal region has a decreased volume. The diaphyseal portion of the stem also has a smaller diameter and length and is highly polished. Titanium alloy was improved with the addition of molybdenum, zirconium, and ferrous (iron), reducing Young's modulus to 74–85 GPa. HA coating, manufactured by a Stryker patented process, keeps the same coating thickness but crystallinity has been improved to 98%. Highly cross-linked polyethylene (Duration) liners with metallic or zirconium heads and ceramic on ceramic heads were used as bearing couplings. From September 1999 to December 2013, 1694 patients were operated on; 428 of them were bilateral, bringing the number to 2122 total hip arthroplasties.

A similar surgical technique was used in both ABG models, and only the surgical instruments for acetabular and femoral preparation varied somewhat between them. The same posterolateral approach, intravenous antibiotic prophylaxis (2nd generation cephalosporins), and antithrombotic prophylaxis protocol (low molecular weight heparin) were used in all cases. Over the years, the only significant changes in postoperative management have been a shorter postoperative immobilization and a reduced length in hospital stay.

Regardless of our participation in an international multicenter follow-up study on ABG I outcomes [35], several long-term follow-up studies have been carried out in our department.

A ten-year follow-up study, on 630 ABG I prostheses implanted in 579 patients, was reported [36]. Clinical outcomes were assessed with the Merle D'Aubigne-Postel score [37], and bone was quality scored, on plain preoperative radiographs, according to the modified Singh scale [38]. Different radiographic items were evaluated at the first, fifth, and tenth postoperative years. Description of radiological findings was done according to the Gruen zones [39] in proximal femur and De Lee and Charnley zones [40] in periacetabular bone. Broker scale for heterotopic ossifications was used [41]. Polyethylene wear was assessed with the Livermore method [42], and granulomatous and osteolytic lesions, secondary to wear debris particles, were also examined. Position of the cup in relation to the anatomic hip rotation centre, cup inclination (opening) angle, and size of the stem in relation to the diameter of the femur were studied too.

On the other hand, 196 ABG II arthroplasties, implanted in 168 patients, were followed up for a mean of 11.3 years [43]. In this case, clinical outcomes were assessed with Harris hip score [44] and subjective outcomes with the EuroQolGroup EQ-5D questionnaire [45]. The Livermore method [42] was used again to evaluate polyethylene wear, even though evaluation was done by means of a computer program since digital radiology had become available. Granulomatous and osteolytic lesions were measured, in this case, according to the scale proposed by Goetz et al. [46].

Both in the ABG I and in the ABG II studies, a statistical *χ* ^2^ analysis for categorical data and percentages comparison and a Student's *t*-test for means comparison of isolated data or between pairs of related data with Pearson correlation were used. The level of significance was set at *P* < .05.

To assess the femoral remodeling changes which occur after stem implantation, a group of patients with ABG I implants had DXA exams which were recorded in the preoperative and throughout the follow-up period (15th day, 3rd, 6th, and 12th month, and annually until the 10th postoperative year) [47]. Similarly, another group of patients with ABG II implants had DXA exams throughout a five-year follow-up period [48].

Finally, simulations were made with the ABG I and ABG II stems, by means of the finite element method, to assess the biomechanical changes which occur in the femur after stem implantation. Simulation results were compared with their respective DXA studies in each model [49–51].

## 3. Results

The gender distribution in the ABG I group was 55.39% male, with a mean age of 58.10 years, and 44.61% female, with a mean age of 61.32 years. In the ABG II group, 70.83% were men and 29.17% were women, and the mean age was 11.26 ± 58.84 years (SD) with a range of 23–77 years.

Clinical outcomes in each implant group are specified below: in the ABG I group the mean preoperative Merle D'Aubigne-Postel score was 7.91, and it increased to 16.21 (range 9–18) at the 10th year; subjective assessment was excellent or good in 82.1% of cases. In the ABG II group, the mean preoperative Harris hip score was 32.55, and the average postoperative score rose to 85.80 (range 26.05–95.82); subjective assessment was excellent or good in 90.32% of cases.

ABG I implants survival at 10-year follow-up was 97.1%. Although all acetabular components were stable, 1.35% of these patients needed revision surgery because of an excessive polyethylene wear. In these cases, the liner was replaced by a highly cross-linked polyethylene, and femoral and/or periacetabular osteolytic lesions were cleaned and grafted. But the prosthetic cup remained stable in all cases and was not replaced.

At 17-year follow-up with ABG I, 18 patients needed revision surgery for major acetabular and/or femoral osteolytic lesions. In such cases both the stem and the cup remained stable; therefore only polyethylene liner was replaced and osteolytic lesions were curetted and grafted. At 20-year follow-up, 21 patients needed revision surgery for major acetabular and/or femoral osteolytic lesions. Only in three patients a replacement of the acetabular cup and femoral stem was performed, implanting a cemented prosthesis in all of them. In the remaining 18 the implants were stable despite osteolytic lesions; therefore only polyethylene liner was replaced and osteolytic lesions were curetted and grafted (Figures 2 to 5).

ABG II prosthesis survival at a mean of 11.3 years of follow-up was 98.30%, with all acetabular components being stable and with no signs of migration.

The key difference between the two model outcomes is polyethylene wear. Duration polyethylene, used in the ABG II model, has shown a 54.55% less wear rate than conventional polyethylene used in the ABG I model. The ABG I polyethylene wear has been greatest in acetabular cups placed in a low position (*P* = .038), with opening angles greater than 46°, and in patients under the age of 65. At ten years of follow-up, the incidence of periacetabular granulomatous lesions in the ABG I group was 44.23% in zone I, 37.11% in zone II, and 15% in zone III; and it was 78% in Gruen zone I and 91.73% in Gruen zone 7. Despite this, all the acetabular and femoral components were stable, even though some stems showed some subsidence. In the ABG II group, granulomatous lesions were very small and only occurred in metal on polyethylene or zirconium on polyethylene couplings. In this group, 9.52% of cases showed osteolytic lesions in acetabular zone I and 12.7% in Gruen zones 1 and 7. Decreased incidence of osteolytic lesions in the ABG II model is due to the lesser wear of the new polyethylene but, in our opinion, the sealing of unused cup holes may also have played a role.

Stem subsidence has been evaluated in both models and significant differences have been found. In the ABG I group, of the cases in which the size of the stem was deemed appropriate, mean subsidence was 1.51 mm at the first year and increased to 3 mm at the 10th year. However, when the size of the stem was deemed large, mean subsidence was 2.29 mm at the first year and reaches 4.17 mm at the 10th year. In the ABG II group, lesser subsidence has been found among the cases in which the size of the stem was deemed appropriate; mean subsidence at the first year was 0.514 mm and rose to 0.638 ± 0.180 (SD) at the end of follow-up, but oversized stems showed 2.435 mm and 2.830 mm, respectively. In both studies oversized stems were associated with a significantly greater subsidence (*P* = .0001).

Femoral remodeling has also shown to be significantly different between the two groups. Up to 90% of cases in the ABG I group showed evident bone devitalization in Gruen zones 1 and 7, while bone loss was less marked in the ABG II group in which it was only detected in 42.07% of cases. Cancellous bone densification in zones 2 and 6 of Gruen was present in 89.42% and 83.26% of cases in the ABG I group, respectively, while in the ABG II group this finding was detected in zone 2 in 34.43% of cases and in zone 6 in 29% of cases. Cancellous bone densification is associated with larger stems (*P* = .002). The high rates of devitalized bone in zones 1 and 7 are caused by the stress-shielding effect which occurs after insertion of a femoral stem. Stress-shielding in femoral zones 1 and 7 is strongly associated with females (*P* = .001), older age (*P* = .001), and low preoperative Singh index (*P* = .001) in both stem models. Comparisons of DXA studies at five-year follow-up show a 13.07% bone loss in zone 1 and 37.5% in zone 7 in the ABG I group, while in the ABG II group the results are 9.07% in zone 1 and 23.88% in zone 7 (Figure 6). These data may mean that design changes in the ABG II stem have achieved a better load transmission.

## 4. Discussion

Our 23 years of experience in routine use of HA-coated hip prostheses is quite satisfactory as regards the long-term stability of implants, in agreement with Geesink [52]. Primary implant stability is favored by HA coating, which provides improved contact between bone and implant [26, 52–56], and osteointegration of HA-coated implants has been sufficiently demonstrated in many studies [26–31, 33, 34]. Through the years, as resorption of the HA coating is caused by chemical dissolution or osteoclastic action, new bone formation replaces it in a percentage which could rise to 78%, according to a number of publications [26, 27, 30, 31, 33, 57]. It is clear, however, that HA-coated implants achieve a stable fixation despite osseointegration not being complete. Moreover, it is well documented that HA debris particles cause no osteolytic reaction [21, 28, 30, 57]. In our personal experience no osteolytic reaction was detected along more than 23 years.

The most important problem we have experienced with the ABG I model is excessive wear of conventional polyethylene and subsequent periprosthetic osteolysis (Figures 7 and 8), although fortunately implants remained stable at 20 years of follow-up. Concerning the ABG II model, with Duration highly crosslinked polyethylene, it has shown much lower wear rates and osteolityc lesions have been significantly less frequent. We believe that sealing unused cup holes has limited the migration of wear debris to acetabular bone, helping to reduce the incidence of osteolytic acetabular lesions. Good peripheral osseointegration of the cup could also have acted as a barrier to wear debris migration [58]. The lower incidence of osteolytic lesions that we have also found in the femur can be explained by the reduced rate of wear debris particles in the ABG II model. But in addition, changes in design of the stem and improved HA crystallinity could have played a role in enhanced osseointegration, which would prevent debris migration into the femoral implant-bone interface [59].

Concerning loads acting on the hip, there are previous works [60, 61] that include a comparative analysis for different combinations of muscle loads, concluding that the more appropriate cases are those that consider the load comprising gluteus medius, iliotibial tract, and psoas iliacus, or only the action from abductor muscle, which produce compression in the femur. For the simulations carried out by our group, the last option was chosen in accordance with the majority of authors [62–65]. Orthoload's database values were used to apply hip reaction forces at the head of the stem and abductor, respectively [66].

Hip arthroplasty modifies the initial tensional state of the hip joint. In the healthy femur, loads are transferred from the femoral head to the lesser trochanter which distributes the compressive forces to the femoral diaphysis [30]. Load distribution can explain the anatomical structure of the primary trabecular bundles of the healthy femur: the arch shape, formed by traction forces, and the principal compression group of Delbet, formed by compression forces [31]. Despite this load pattern is inverted after hip replacement, so that the stresses are transferred fundamentally from the prosthetic head to the stem, which transmits mechanical loads to the zone of the femur corresponding with the end of stem HA coating. Thus, a bottleneck effect is produced, as was demonstrated in the simulation (Figure 9), which leads to stress-shielding. Due to these changes in the transmission of forces all implants cause remodeling changes in the proximal femur, though cemented stems do it to a lesser extent [67]. Adaptative remodeling is due to an alteration in loads transmission produced by the femoral stem. It is regulated by Wolf's Law [67, 68] and is a multifactorial process influenced by the bone quality and stiffness, implant design and stiffness, type of bone fixation, and forces acting on the femur [64, 69–75]. As Huiskes et al. [68] pointed out, preoperative bone mass of the proximal femur is a very important factor in adaptative remodeling. ABG stems theoretically have a metaphyseal anchorage and, like other similar designs, were intended to transmit loads from proximal to distal femur and avoid stress-shielding. But so far, this goal has not been achieved as McAuley et al. [76] demonstrated. Loads are mostly transmitted through the distal end of the metaphyseal bone, right where stem coating ends. Lack of loading on the proximal femur is a common problem to all anatomical stem designs [77–79]. The biomechanical finite element (FE) studies we have conducted on both ABG stems [49–51] support this assertion (Figure 9). The highest incidence of cancellous bone densification and cortical bone sclerosis detected in zones 2 and 6 of Gruen, in oversized stems, is explained by the tight fit of the implant into the medullary canal, which causes higher stresses in these zones (Figure 10).

Correlation between the data obtained from finite element simulations and those obtained from DXA with ABG I at 10 years [47] and ABG II at 5 years [48] shows that the ABG-II stem is more effective than the ABG-I model, because the former generates higher tensional values on femoral bone, resulting in lesser bone loss (Figure 6). Thus, improved loads transmission matches biological findings obtained with DXA. We believe that the design and the alloy of stem have major importance in the transmission of loads in the femur. Changes in the lateral metaphyseal area and shoulder of the ABG II with a more trapezoidal (tapered) design have possibly contributed to improving the transmission, which is in accordance with the experience of Leali and Fetto with a lateral flare stem [80].

On the other hand, the lower length and volume of the ABG II stem allow us to better preserve the cancellous bone in the proximal femur which is an important factor for adaptive remodeling after implanting a femoral stem [67]. The decrease in volume of the metaphyseal area of stem ABG II has not affected the primary and secondary stability thereof, as shown by the values of mean subsidence in ABG II rods, which are 78.73% lower than the corresponding to the ABG I stem, confirming the effectiveness of design changes.

Adaptative remodeling and loads transmission influence the replacement of HA coating by new bone. Osseointegration rate is higher in heaviest loaded areas according to Wolf's law [26], which is supported by our findings: increased osseointegration in the metaphyseal-diaphyseal transition area and persistence of HA coating in the proximal metaphyseal area for more than 8 years after implantation of the stem [31].

A good preoperative planning [79] and meticulous surgical technique is needed in cementless hip arthroplasty to achieve a perfect press-fit of implants which provides an adequate primary fixation. Acetabular reaming must progress carefully down to bleeding subchondral bone, which is essential for secondary fixation, that is, osseointegration [81]. A similar technique should be used in femoral preparation. HA-coated implants require the same careful technique because HA coating does not solve technical errors. Critical analysis of our experience makes us understand that we have made incorrect indications in older patients with poor bone quality, who required oversized stems resulting in significant subsidence. Therefore, we reaffirm that appropriate indication and preoperative planning are essential requirements for good outcomes. Although design improvements in the ABG II stem have led to a decreased incidence of stress-shielding and subsidence, we have to bear in mind that bone mass index is critical to minimize stress-shielding, as Huiskes et al. [68] noted. The new Duration polyethylene has decreased wear by 54.55% compared to the conventional one, but alternative bearing surfaces should be considered in young patients with more demanding physical activity (ceramic-ceramic, in which we observed no measurable wear over an 11-year follow-up period).

Our HA-coated hip implants series has high long-term survival, in line with other author series [34, 59, 77, 82–96]. The excellent stability of HA-coated implants has been demonstrated even in elderly patients [97]. Other studies find no advantage in HA-coated implants over metallic-coated designs, mainly in the acetabular cups [98–104]. Some even believe that HA coating is a risk factor which contributes to loosening and is associated with poor long-term results in acetabular cups [105] in the HA coating stems, finding no advantage over metallic-coated implants [106]. We think it is risky attributing the mobilization of acetabular cups only to the possible delamination of the HA, and the consequent release of particles, when it coexists with excessive polyethylene wear in these cases, which we consider primarily responsible for osteolytic lesions. In our experience with the ABG I prosthesis, which presents an excessive polyethylene wear, 21 patients with 20-year follow-up needed major revision surgery for acetabular and/or femoral osteolytic lesions. The replacement of the acetabular cup and femoral stem was performed only in three patients; the rest had perfect stability of their implants, demonstrating the advantages of HA coating for reaching an excellent osseointegration. The data of Danish Hip Arthroplasty Registry show excellent medium-term survival of HA-coated and non-HA-coated implants [107] and the data of the Finnish Arthroplasty Register showed a better survival of HA-coated implants in young patients [108]; the Norwegian Arthroplasty Register showed that one brand of HA-coated stem had better survival than some non-HA-coated components [109]. Our wide and long-term experience in HA-coated hip implants and our outcome with excellent survival go against these assertions, in agreement with many authors [34, 59, 77, 82–96], but HA is not a magic powder [89] and the indication and surgical technique must be careful and correct in the HA-coated prostheses.

The survival of HA coated acetabular cups is better than of cemented cups especially in younger people which have a high percentage of long-term loosening, while the long-term survival of cemented stems reaches 85–95% according to papers published, depending on follow-up time, cementing techniques, and patient age [107–118]. Our personal experience with cemented hip prosthesis has similar survival rates. Survival of cementless HA-coated prostheses is superior in the acetabular components to the published results of cemented prostheses [59, 77, 83–91] and it is comparable in the femoral stems. Moreover if in the long term it is necessary to perform a replacement this will be technically easier in cementless prostheses because we will have more bone stock for future revision surgery, considering that today hip arthroplasties are implanted at very young patients with high functional demands [119–121] that possibly will need in the long term this type of surgery.

In conclusion, HA-coated hip implants are a reliable alternative, mainly in young people, which can achieve long-term survival provided that certain requirements are met: good design selection, sound choice of bearing surfaces based on patient life expectancy, meticulous surgical technique, and indications based on adequate bone quality.

## Figures and Tables

**Figure 1:** (a) ABG-I stem and acetabular cups; (b) ABG-II stem and acetabular cup.

**Figure 2:** X-ray image of patient with follow-up at 12 y. Osteolysis in acetabulum produced by excessive polyethylene wear.

**Figure 3:** Computed tomography of the same case in Figure 2. Osteolysis in acetabulum.

**Figure 4:** X-ray control of patient in Figures 2 and 3, after 4 y follow-up, after changing polyethylene and fulfilling with bone graft the acetabulum osteolysis. No change of original implant.

**Figure 5:** Same case as in Figures 2, 3, and 4. X-ray control image in 2013, after 8 y. follow-up of second surgery with original implant since 1993.

**Figure 6:** Evolution of bone mass density for ABG I (blue) and ABG II (red), corresponding to five-year follow-up, in the Gruen zones.

**Figure 7:** X-ray image of patient with follow-up at 12 y. Excessive polyethylene wear. Osteolysis in metaphyseal of femur.

**Figure 8:** Same case as in Figure 7, after changing polyethylene and fulfilling with bone graft and femoral mesh. No change of original implant. Control at 20 y. of primary surgery.

**Figure 9:** Maximum and minimum principal stress flow in the models with prosthesis (from a FE simulation).

**Figure 10:** X-ray image of oversized stem in right femur with cancellous bone densification in support area (zone A) and bone resorption (zone B).

## Abbreviations

HA: Hydroxyapatite
ABG: Anatomique benoist giraud
DXA: Dual-emission X-ray absorptiometry
FE: Finite elements.
